# Application of a FL Time Series Building Model in Mobile Network Interaction Anomaly Detection in the Internet of Things Environment

**DOI:** 10.1155/2022/2760966

**Published:** 2022-02-01

**Authors:** Haotian Chen, Sukhoon Lee, Dongwon Jeong

**Affiliations:** ^1^College of Information and Engineering, Hebei GEO University, Shijiazhuang 050031, China; ^2^Department of Software Convergence Engineering, Kunsan National University, Gunsan 54150, Republic of Korea

## Abstract

With the continuous development of the social economy, mobile network is becoming more and more popular. However, it should be noted that it is vulnerable to different security risks, so it is extremely important to detect abnormal behaviors in mobile network interaction. This paper mainly introduces how to detect the characteristic data of mobile Internet interaction behavior based on IOT FL time series component model, set the corresponding threshold to screen the abnormal data, and then use K-means++ clustering algorithm to obtain the abnormal set of multiple interactive data, and conduct intersection operation on all abnormal sets, so as to obtain the final abnormal detection object set. The simulation results show that the FL time series component model of the Internet of Things is effective and can support abnormal detection of mobile network interaction behavior.

## 1. Introduction

With the continuous development of social economy, internet technology and mobile network are gradually improved, the corresponding mobile hardware devices are constantly upgraded and updated, and the interaction behavior of devices is also constantly frequent [1–3]. Among various behaviors of mobile network interaction, it is vulnerable to diversified attacks. Once abnormal behaviors of mobile network interaction occur, they often cause many adverse effects on network devices [4–6]. In addition to the attacks on the network, there are also attacks on the devices of the Internet of Things [7]. As IoT devices can generate high-dimensional data with obvious characteristics, such as temperature measurement, video monitoring, and water level telemetry, IoT devices have been deeply applied in many aspects [8, 9]. The interaction of mobile network is mainly aimed at interaction behavior, because the interactive network is easy to accept, simple to operate, and so on and has been applied in many computer networks, bringing a lot of mobile network interaction behavior [10, 11].

Therefore, how to effectively identify abnormal behavior and distinguish normal mobile network interaction is worth studying. Scholars in the industry classify data samples of interactive behaviors through support-vector machines, realize linear transformation, and judge and identify them according to the final results. Some scholars use a genetic algorithm to build a detection model to realize the aggregation of interactive behavior for overall anomaly detection. In addition, specific classification of abnormal behaviors is realized based on the discrimination of abnormal data by the wavelet model [10, 12, 13]. However, these methods have certain limitations, especially in feature extraction and direction recognition, which are difficult to be finely divided [14].

According to these limitations and demand, this study is based on the Internet of FL classification model and time series data of mobile network interaction behavior characteristics, given the corresponding detection threshold detecting abnormal behavior, to test the different interaction behavior characteristics, get different behavior characteristic collection, and finally extract the corresponding mobile network interaction behavior anomaly detection, to remove the corresponding dangerous network threats, aiming to improve the security and reliability of mobile network.

## 2. FL Time Series Component Model of Internet of Things

For the FL time series component model of the Internet of Things, it is necessary to classify all the data first and select the corresponding component model. But not for the model, a model for all the analysis of the situation, different simulation component model, is only able to reflect the data collection of now, cannot fully reflect all the law, and therefore, can only from the perspective of a different combination of the corresponding model, using comprehensive consideration, to maximize the analysis of existing data, in order to further improve the corresponding analysis results [14, 15].

The corresponding mobile network time series as is set as{*x*_*t*_, *t*=1,2, *L*}, and the mobile interaction volume (*x*_*n*_ is the real value) of the existing time period N is analyzed. If K analysis methods (*K* ≥ 2) are selected, the predicted result value of method I can be represented by *f*_*ni*_=*x*_*n*_ − *f*_*ni*_(*i*=1,2, *L*, *K*).

Through the analysis and simulation of time period N, it can be calculated by

(1) $$\begin{array}{c} x_{n}^{\text{\$}}=f_{n}=\overset{k}{\underset{i=1}{\sum }}w_{i}f_{ni}, \end{array}$$

where *w*_*i*_ (*i*=1,2, *L*|, *K*, and ∑_*i*=1_^*k*^*w*_*i*_=1) is the combined weight of the i-th method.

Generally speaking, for a combined component model, as submodels are different, it is necessary to conduct a comprehensive analysis of the proportion of the combined model. The combined model needs to conduct analysis and simulation based on actual data and select different weight values according to different data feature sets to ensure that the analysis model is more effective [16, 17].

### 2.1. Time Series Model

The so-called time series model is the practice sequence model [18, 19], which sorts the practice sequence to form a continuous time axis. By analyzing the changes in the time axis, the trend, possibility, and effect of the existing data can be judged. Depending on the data objects analyzed, they can include moving averages and exponential smoothing. For the time series component model, its specific calculation is shown in the following formula:

(2) $$\begin{array}{c} s_{t+1}=\alpha x_{t}+\left(1-\alpha \right)s_{t}=s_{t}+\alpha \left(x_{t}-s_{t}\right), \end{array}$$

where *α* is the coefficient and *x*_*t*_ − *s*_*t*_ is the error of the previous forecast.

From the perspective of component model analysis, the closer the analysis result is to the observation value, the better the analysis effect is, so the selection of the component model is extremely important.

### 2.2. FL Model

Based on the time series model, this study proposes an FL model for mobile network interaction by integrating support-vector machine classification and genetic algorithm classification algorithm. The specific framework is shown in Figure 1.

The Jordan network is adopted to establish the prediction model, and the output function is shown in the following formula:

(3) $$\begin{array}{c} f_{n}\left(t\right)=\sum_{i=1}^{q}w_{i}\phi_{i}\left(t\right)+b\left(t\right), \end{array}$$

where input and output weight values are represented by *ϕ*_*i*_(*t*); the output function of the hidden layer is represented by *f*_sfg_′. Its specific calculation is shown in the following formula:

(4) $$\begin{array}{c} \phi =g\left(\sum_{j=1}^{p}v_{ij}x_{j}\left(t\right)+\sum_{k=1}^{s}\sum_{v=1}^{r}w_{ikv}f_{v}.\left(t-k\right)+b_{i}\left(t\right)\right), \end{array}$$

where the weight value between the input layer and the hidden layer is represented by *v*_*ij*_. The weight of *k* delay between connecting layer and hidden layer is represented by *w*_*ikv*_. The weight value is adjusted and improved according to the neural network, and the specific algorithm is shown in the following formula:

(5) $$\begin{array}{c} f_{n}\left(t\right)=h\left(x^{T}\left(t\right)\Phi \left(t\right)\right), \end{array}$$

where *h*(.) is the nonlinear function of *x*^*T*^(*t*) and *f*_*n*_(*t*); input variable *x*^*T*^(*t*)=[*x*_1_(*t*), *L*, *x*_*p*_(*t*)]^*T*^; and the weight vector Φ(*t*)=[Φ(*t*), *L*, Φ_*p*_(*t*)].

The predicted network transmission amount at the predicted time is shown in the following formula:

(6) $$\begin{array}{c} f=\sum_{i=1}^{p}W^{T}\psi \left(x^{T}\left(t\right)\right)+b\left(t\right). \end{array}$$

### 2.3. Constraint Test

For abnormal data prediction results that cannot be determined where the specific occurrence of abnormal data occurs, by constructing an F statistic based on the proportional relationship of the abnormal data measurement value, and combining it with the abnormal data-constrained residual statistic, and the occurrence of abnormal data in the steady-state process of preliminary detection of the error of the wavelet amount.

The data containing n' interactive abnormal behaviors are measured, the corresponding number of nodes is set as P, and the specific residual constraint measurement is calculated using the following formula:

(7) $$\begin{array}{c} e=n^{\prime }P \end{array}$$

where interaction behavior constraints of mobile network are represented by *A* (*P* × *n*), corresponding statistics are established, and the following formula is used for calculation:

(8) $$\begin{array}{c} Z_{j}=\frac{e_{j}}{\sqrt{v_{jj}}}. \end{array}$$

According to formula (8), it can be seen that within the range of *z*_*j*_ : *N*(0,1), the abnormal data detection level can be set as *α*, and the detection critical point *Z*(*a*/2) can be determined. If the condition (|*Z*_*J*_| > *Z*(*a*/2)) is met, it is considered that the jth abnormal data are incorrect, and there is also a wavelet error in one or more data values associated with it.

### 2.4. Coordinate and Sort Out Error Data

The abnormal detection of mobile interaction behavior is determined based on the detection of the targeted data, and the spatiotemporal correction of the abnormal behavior data is carried out from the spatiotemporal perspective to obtain the corresponding abnormal behavior data. The specific calculation is shown in formulas (9) and (10):

(9) $$\begin{array}{c} x^{\%}=x^{\prime }+a, \end{array}$$

(10) $$\begin{array}{c} \Gamma \left(x^{\prime },U\right)=0, \end{array}$$

where the mobile interaction behavior is represented by *x*^*o*^, the data to be tested are set as U, and the function vector is represented by Γ. The specific calculation is shown in the following formula:

(11) $$\begin{array}{c} \min\sum_{i=1}^{n}\frac{\left(x_{i},x_{i}\right)}{\sigma_{i}^{2}}, \end{array}$$

where the coordination value of a set of corrected wavelet error detection data is represented by *x*_*i*_^$^, and the measurement covariance is represented by *σ*_*i*_. The formula (11) is converted to :

(12) $$\begin{array}{c} \min\left[{\left(\mu -x\right)}^{T}Q^{-1}\left(\mu -x\right)\right], \end{array}$$

where focusing element is represented by *Q*, and linear constraint solution can be expressed by

(13) $$\begin{array}{c} \min\left[\left(\mu -x^{\prime }\right)Q^{-1}\left(\mu -x^{\prime }\right)\right]. \end{array}$$

First, a Lagrange function is defined, and then, the Lagrange method is used to solve it, as shown in the following formula:

(14) $$\begin{array}{c} L=\left(\mu -x^{\prime }\right)Q^{-1}\left(\mu -x^{\prime }\right)-2\lambda \left(A\right). \end{array}$$

In the formula, *λ* is the multiplier vector of Lagrange so that the equation of partial derivative obtained is zero, as shown in the following formula:

(15) $$\begin{array}{c} \frac{\partial L}{\partial U}=2Q^{-1}\left(\mu -U\right)-2A\lambda =0. \end{array}$$

According to formula (15), the unmeasured data are solved and the formula is further simplified, as shown in the following formula:

(16) $$\begin{array}{c} U={\left(B^{T},QB\right)}^{-1}B^{T}Q^{-1}\left(\mu \right). \end{array}$$

After solving the *B*^*T*^ matrix, if the inverse matrix does not exist, the equation system has no solution. At this time, all network measurement data must be calibrated, all untested interactive network measurement data variables can also be estimated as Yes, only when these conditions are met, and the A and B matrices can be inverted. For the inestimable or uncorrectable interactive network measurement data, the projection matrix method can be used to eliminate it.

According to the above steps, the accurate detection of the abnormal data of the interactive network is completed.

### 2.5. System Principle of Abnormal Data Accurate Detection of Mobile Network Interaction Behavior

During the operation and implementation of mobile network, there are often external interference and threats, and more abnormal behavior data are prone to appear. To detect abnormal data, a detailed analysis of interaction behavior is required, and the specific steps mainly include the following.

The phase space reconstruction theory is used to normalize the original interactive network data, and the normalized network data are reconstructed in phase space. According to the FL criterion, the linear regression problem of abnormal data training samples is converted into a constrained secondary optimization problem, and the least-squares support-vector machine nonlinear model of the current time series is obtained, thereby completing the preliminary detection of abnormal data.

The delay coordinate is used to carry out the spatial emphasis of network time series, and the specific calculation is shown in the following formula:

(17) $$\begin{array}{c} X\left(n\right)=\left[x\left(n\right),L,x\left(n-\left(m-1\right)T\right)\right], \end{array}$$

where *m* is the measurement standard value of interactive network time series data, and *T* is the measurement time. It is supposed that *F*(.) represents the interactive network time series prediction data model. For the linear regression problem of *n* network data, (*x*_*i*_, *y*_*i*_, ) can be set as the detection dataset, *x*_*i*_*ɛR*^*d*^ is the input mode of the i-th abnormal data training sample, and *iɛR* corresponds to the expected output of the i-th data. The linear regression function can be expressed by the following formula:

(18) $$\begin{array}{c} y\left(x\right)=w^{T}x+b, \end{array}$$

where the specific classification surface is represented by *b*, and the partial derivative is represented by *w*. According to the corresponding optimal solution, the specific solution is shown in the following formula:

(19) $$\begin{array}{c} \min J\left(w,\xi \right)=\frac{1}{2}w^{i}w+\frac{\gamma }{2}\sum_{i=1}^{n}\xi_{i}^{2}. \end{array}$$

Constraint conditions can be calculated by

(20) $$\begin{array}{c} y_{i}=w^{T}x_{i}+b+\xi_{i},i=1,L,n, \end{array}$$

where tunable parameters are represented by *r* > 0. The specific available formula is as follows:

(21) $$\begin{array}{c} L\left(w,b,\xi ,a\right)=\frac{1}{2}w^{T}x_{i}+\sum_{i=1}^{n}\xi_{i}^{2}-\left(b+\xi_{i}-a_{i}\right). \end{array}$$

LS-SVM linear regression equation can be obtained as shown in the following formula:

(22) $$\begin{array}{c} f\left(x\right)=\sum_{i=1}^{n}a_{i}\left(x_{i}^{T},x\right)+b. \end{array}$$

Based on formula (22), the LS-SVM nonlinear regression equation can be further solved as

(23) $$\begin{array}{c} f\left(x\right)=\sum_{i=1}^{n}a_{i}K\left(x_{i},x\right)+b. \end{array}$$

To detect abnormal mobile network interaction behavior based on Internet FL time series, it is necessary to first extract the features of high-dimensional data components to accurately achieve detection effectiveness, and then set corresponding thresholds, use abnormal data aggregation, and perform data based on corresponding random mapping algorithms. When the data do not conform to the corresponding aggregation, the intersection operation of all abnormal data is needed to obtain the corresponding anomaly detection. The specific process is shown in Figure 2.

## 3. Feature Extraction of Network High-Dimensional Data Time Series Components

First, according to the different components of the high-dimensional data time series in the current mobile network, the characteristics of the existing data components are adjusted. The specific method is to extract the time series components of the current network high-dimensional data and solve the actual eigenvalues and eigenvectors of the covariance matrix of the data samples, including the calculation of the inner product of the data vector. The following gives the direction vector of the current network high-dimensional data time series in the feature space mapping. The specific steps are as follows:

Let *μ*_sert_′ represent the time period component characteristics of the mobile interaction data, *d*_dgj_′ represent the highest time series pattern of the current data, and *F*_*A*_ represent the linear fitting function of the data currently interacting with the time series data matrix A.

The corresponding formula is used to carry out mobile network interaction and extract high-dimensional data components, as shown in following formula:

(24) $$\begin{array}{c} E_{\text{drp}}^{\prime }=\frac{A⊕F_{A}}{d_{\text{dgj}}^{\prime }}\pm \left\{\mu_{\text{sert}}^{\prime }\mp l_{\text{fty}}^{\prime }\right\}. \end{array}$$

For nonrepetitive data, the following formula is used to calculate the maximum component characteristics of the data:

(25) $$\begin{array}{c} R_{\text{kptce}}^{\prime }=\frac{R_{SE}^{\prime }\mp R_{\text{kwe}}^{\prime }}{B_{\text{drty}}^{\prime }}l_{\text{fty}}^{\prime }\mp \left\{f_{\text{sf}g}^{\prime }\pm d_{\text{dhk}}^{\prime }\right\}. \end{array}$$

Second, the following formulas are used to solve data samples:

(26) $$\begin{array}{c} R_{\text{drty}}^{\prime }=\frac{\Phi_{fh}^{\prime }⊕x_{\text{sfkp}}^{\prime }}{e_{\text{sgw}}^{\prime }\pm r_{ry}^{\prime }}\mp \left\{N\pm s_{\text{sgj}}^{\prime }\right\}, \end{array}$$

(27) $$\begin{array}{c} P_{\text{dfty}}^{\prime }=\frac{\Phi_{fh}^{\prime }⊕x_{\text{sfkp}}^{\prime }}{e_{\text{sgw}}^{\prime }\pm r_{ry}^{\prime }}\mp \left\{\frac{N\pm s_{\text{sgj}}^{\prime }}{R_{\text{dfty}}^{\prime }}\right\}. \end{array}$$

According to formula (28), the single direction vector formed after the subset space of current mobile network interactive data is mapped to the high-dimensional feature space can be calculated as follows:

(28) $$\begin{array}{c} R_{\text{erp}}^{\prime }=\frac{K_{\text{sgh}}^{\prime }\mp \varpi_{sf}^{\prime }h}{t_{\text{dhj}}^{\prime }\times k^{\prime }}⊗m\frac{sd_{\text{dghj}}^{\prime }}{R_{\text{swekk}}^{\prime }}R_{\text{kkp}}^{\prime }, \end{array}$$

where the Gaussian radial basis kernel function is represented by *K*_sgh_′, and the corresponding vector of the characteristic value of the current interactive data is represented by *h*.

According to the above steps, using the time abnormal point sequence of the current network interaction behavior data, the high-dimensional time data components are determined, the actual eigenvalues of each sequence component are extracted, and the component eigenspace is solved to confirm the eigenvector value of the data under the covariance matrix, in which subsequent mobile network interaction behavior anomaly detection lays the foundation.

### 3.1. Setting Detection Thresholds

Taking the previously obtained mobile network interaction behavior data feature value subset and the forward vector data of the high-dimensional feature space as the core, a constant deviation function is set up, the detection fitting error under different interaction behavior data is calculated, and the minimum value of the deviation function is solved. This value is the abnormal value of the current interactive high-dimensional data. Using this threshold, a random mapping can be established to complete anomaly detection. The specific steps are as follows.

Assuming that *I*_fty_′ represents the nonlinear restoring force of interactive data in the current IoT network environment, *σ*_ser_′ represents the data chaotic transition period, and *η*_awer_′ represents the nonlinear restoring force of the current interactive behavior data. *η*_awer_′ is divided into multiple segments and *d*_*gh*_′ segments, based on the direction vector of the extracted interactive data subset mapped to the high-dimensional feature space.

The following formula is used to calculate data deviation:

(29) $$\begin{array}{c} T_{\text{wer}}^{\prime }=\frac{d_{gh}^{\prime }\times \eta_{\text{awer}}^{\prime }}{d_{gh}^{\prime }}. \end{array}$$

It is assumed that *ε*_fty_′ represents the fitting error of abnormal interactive data at the end of different time series, which can be calculated by

(30) $$\begin{array}{c} \varepsilon_{\text{fty}}^{\prime }=\frac{U_{\text{sert}}^{\prime }\times h\times T_{\text{wer}}^{\prime }}{g_{\text{fjp}}^{\prime \prime }}. \end{array}$$

In formula (30), *U*_sert_′ represents the fixed segment of the current mobile network time series and *T*_*wer*_′ represents the actual deviation of *U*_sert_′ under the fixed segment.

The following formula is used to calculate the corresponding deviation of the abnormal function of the current interaction behavior:

(31) $$\begin{array}{c} Q_{\text{ser}}^{\prime }=\frac{\gamma_{\text{frt}}^{\prime }\times T_{\text{wer}}^{\prime }}{p_{\text{fyu}}^{\prime }}\pm R_{\text{llp}}^{\prime }. \end{array}$$

In formula (31), *p*_fyu_′ represents the deviation amount of data points of abnormal network interaction behavior, and *R*_llp_′ represents the interaction time series of the actual segmented function.

Let *ξ*_*kp*_′ represent the actual number of current data points, and then, the following formula is used to determine the data detection threshold:

(32) $$\begin{array}{c} R_{\text{werk}}^{\prime }=\frac{\xi_{kp}^{\prime }\mp Q_{\text{ser}}^{\prime }\mp \varepsilon_{\text{fty}}^{\prime }}{T_{\text{wer}}^{\prime }}. \end{array}$$

### 3.2. Building Random Mappings

By detecting thresholds, random mapping can be established to complete high-dimensional matching.

The hash value is calculated as shown in

(33) $$\begin{array}{c} h_{a,b}\left(\text{port}\right)=\left[\left(ak+b\right)\mathrm{mod}p\right]\mathrm{mod}M. \end{array}$$

In the formula, *a*, *b* ∈ {0,1, ⋯, *p* − 1}, according to the range comparison, the final hash value falls between 0 and m-1.

The establishment of the hash function is shown in the following formula:

(34) $$\begin{array}{c} h_{a}\langle a_{1},a_{2},a_{3},a_{4}\rangle =\left(a_{1}x_{1}+a_{2}x_{2}+a_{3}x_{3}+a_{4}x_{4}\right)\mathrm{mod}M. \end{array}$$

In the above function, low collisions of N random mappings can be guaranteed. At this time, the interactive data collisions will show a decreasing trend with the mapping value. At this time, the K-means++ algorithm is introduced in conjunction with the mapping value. The framework of this algorithm is a characteristic clustering algorithm. The basic principle of determining the clustering center is that the initial clustering of interactive data needs to be as wide as possible. Then, the steps for establishing interactive mapping random data are summarized as follows:

  Step 1: according to the Internet of Things database, multiple time series datasets are input, and one as the data center is randomly selected
   Step 2: for any point *x* on the current dataset, the distance *d* from the cluster center is calculated
   Step 3: a new interactive data point is selected as the cluster center, and its selection condition is as follows: the point with the largest distance
   Step 4: steps 2 and 3 above are repeated until multiple cluster centers are determined, and the total number is K
   Step 5: data clustering is performed, the sum of d1 and d2 is calculated, it is recorded as Sum, and the K value is looped through to complete the clustering

### 3.3. Realizing Interactive Anomaly Detection

The core of anomaly detection is to use the random mapping and clustering established above to obtain the detected abnormal value SON (sketch output number) of the current mobile network interaction data, perform data reverse analysis on the current SON value according to the abnormal mapping rules, and finally obtain the source of the interaction anomaly IP address to realize anomaly detection. The specific process is as follows: first, random mapping of the current Internet of Things interaction to the source IP is performed, and the SON value corresponding to all the source IPs is obtained. Then, the various interactive data objects corresponding to the IP are continuously clustered at the global mapping level to obtain multiple SONs. Data sequence time feature package and the calculation of the feature package dimension need to be based on the abovementioned feature dimension vector and vector, and in addition, the SON value at the same time needs to be quantitatively weighted.

After completing the above steps, the time reports of multiple SON data sequences are formed into an *X* matrix, and the current mobile network interactive data are unsupervised clustering detection.

First, the parallel time axis *T* is used to intercept the overall timing S of the current mobile network to ensure the real-time performance of the current detection, so as to obtain the clustering times as shown in the following formula:

(35) $$\begin{array}{c} C=\frac{S}{T}. \end{array}$$

In particular, according to the current hash operation rules of *n* times, the outliers corresponding to K times clustering results are continuously reversed into IP sets, and the hash of *n* times is obtained after the result union, so as to realize abnormal detection of mobile network interaction behavior. The IP set of the abnormal data source is shown in the following formula:

(36) $$\begin{array}{c} {\text{alarmObj}}_{n}=\overset{c}{\underset{i=1}{\cup }}{\text{alarmObj}}_{n}^{j}. \end{array}$$

## 4. Experimental Simulation

In order to conduct the FL time series component model of the Internet of Things for abnormal detection of mobile network interaction behavior, the corresponding simulation dataset was selected for the test.

### 4.1. Experimental Parameters

According to the data, the formulas defined by TPR and FPR are shown as follows:

(37) $$\begin{array}{c} \text{TPR}=\frac{FP}{FP+TN}, \end{array}$$

(38) $$\begin{array}{c} \text{FPR}=\frac{TP}{TP+TN}, \end{array}$$

where TPR is the current proportion of positive classes and FPR is the current proportion of negative classes.

According to the corresponding simulation experiment, the experimental time scale is established, and the results are shown in Figure 3.

In Figure 3, each data point represents the corresponding relationship between TPR and FPR on the corresponding time scale. The two curves are the function fitting values of TPR and FPR under multiple time scales. It can be seen that as time continues to increase, TPR and FPR both change from large to small and then from small to large, but the general trend is an upward state, and the conversion amplitude decreases. This is because the sudden abnormal flow set by the experimental network will adversely affect the detection. According to the experimental evaluation of the current experimental environment, the optimal base percentage of TPR and FPR is 28.28%.

It can be seen from the results that with the increase in time, TPR and FPR change from large to small but generally show an upward state, and the transformation amplitude decreases and presents a waveform.

Figure 4 shows the time ROC curve under the current base percentage. This curve determines the coherence of experimental network interaction. In ROC characterization, the point close to the upper left corner represents the detection rate of the time scale.

After constructing the interactive time scale, it is necessary to summarize the experimental hash table, as shown in Figure 5.

### 4.2. Detection Comparison

The design takes the traditional support vector machine classifier anomaly detection method as the comparison group and compares it with the detection method designed in this study. The detection target is the real-time index of current interactive data detection.

As can be seen from Figure 6, the abscissa in the figure is FPR and the ordinate is TPR. Two different shape points correspond to two different methods. According to the data standard, it is certain that the denser the data points, the better the real-time performance. It can be seen from the data results that the FL time series component model of the Internet of Things is more effective, making the data points significantly closer.

By comparing the corresponding detection methods, the detection distribution of abnormal data is realized.

It can be seen from the results that the root mean square errors are 0.05 and 0.09, respectively, and the relative errors are 0.03 and 0.07. Therefore, it can be seen that the FL time series component model of the Internet of Things is effective (Figure 7).

Three performance indexes, namely, OP, AVTI, and OPF, are used to test the F statistic method adopted by the proposed method, which is defined by the following formula, such as formulas (39)–(40):

(39) $$\begin{array}{c} \text{OP}=\frac{\begin{array}{c} \text{total number of wavelet errors detected correctly} \end{array}}{\begin{array}{c} \text{number of wavelet errors} \end{array}}, \end{array}$$

(40) $$\begin{array}{c} \text{AVTI}=\frac{\begin{array}{c} \text{total number of wavelet errors detected by error} \end{array}}{\begin{array}{c} \text{number of experiments} \end{array}}, \end{array}$$

(41) $$\begin{array}{c} \text{OPF}=\frac{\begin{array}{c} \text{total number of wavelet errors detected correctly} \end{array}}{\begin{array}{c} \text{number of experiments} \end{array}}. \end{array}$$

The anomaly detection of mobile network interaction behavior is analyzed, and the corresponding confidence is set. The specific evaluation results are shown in Figure 8.

It can be seen from the results in Figure 8 that the FL time series component model of the Internet of Things is effective, the detected abnormal data are 100%, and the performance is relatively reliable.

The proposed method and the other two algorithms are used to accurately detect abnormal data in the interactive network (Figure 9).

It can be seen from the results that the abnormal data detected by the proposed method in unit time is almost consistent with the amount of abnormal data given, which proves that the FL time series component model of the Internet of Things is effective.

## 5. Conclusions

With the continuous development of internet of things technology and 5 G network communication technology, mobile network interaction behavior is becoming more and more frequent. Therefore, the detection of mobile network interaction abnormal behavior is worth focusing on. Based on the FL time series component model of the internet of things, this study summarizes the characteristic data of mobile network interaction behavior, sets the corresponding threshold for data inspection, uses different interaction behaviors for cluster detection, realizes the interactive abnormal dataset, and uses the intersection operation to realize the simulation experiment. The simulation results show that the FL time series component model of the Internet of Things is reliable and can effectively detect abnormal behavior.

## Figures and Tables

**Figure 1:** FL model framework.

**Figure 2:** Detection flowchart.

**Figure 3:** Fitting curve of TPR and FPR under the time scale.

**Figure 4:** ROC curve of time scale.

**Figure 5:** Experimental hash parameters.

**Figure 6:** Relationship between detection results and prediction results of the proposed method.

**Figure 7:** Relationship between detection results and prediction results.

**Figure 8:** Performance evaluation of F statistic method.

**Figure 9:** Detection amount of wavelet data with different methods in unit time.

## Data Availability

Data sharing is not applicable to this article as no datasets were generated or analyzed during the current study.
